# The Diagnostic Value of Contrast-Enhanced Ultrasound and Enhanced CT Combined with Tumor Markers AFP and CA199 in Liver Cancer

**DOI:** 10.1155/2022/5074571

**Published:** 2022-02-21

**Authors:** Yunpeng Kong, Yan Jing, Hongmei Sun, Shisheng Zhou

**Affiliations:** ^1^Department of Imaging, People's Hospital of Rizhao, Rizhao 276800, Shandong Province, China; ^2^Department of Imaging, Zhangqiu District Hospital of Traditional Chinese Medicine, Jinan 250200, Shandong Province, China; ^3^Hospital Infection-Control Department, Zhangqiu District People's Hospital, Jinan 250200, Shandong Province, China; ^4^Department of Ultrasound, Kangtai Hospital, Kangtai 264000, Shandong Province, China

## Abstract

**Background:**

Early screening and diagnosis are of great significance to the treatment and prognosis of patients with liver cancer. This study aims to explore the application value of contrast-enhanced ultrasound and enhanced CT combined with tumor markers alpha-fetoprotein (AFP) and carbohydrate antigen 199 (CA199) in the diagnosis of liver cancer.

**Methods:**

Liver cancer group (*n* = 256), benign disease group (*n* = 110), and control group (*n* = 50) participated in this study. The liver cancer and benign disease groups were diagnosed pathologically by contrast-enhanced ultrasound and enhanced CT before operation. The electrochemiluminescence method was used to detect the content of AFP and CA199. And the receiver operating characteristic (ROC) curve was drawn.

**Results:**

The detection rate of contrast-enhanced ultrasound is higher than that of enhanced CT. Serum levels of AFP and CA199 in the liver cancer group were significantly higher than those in the benign lesion group and the control group. The ROC curve showed that the sensitivity, accuracy, and negative prediction rate of contrast-enhanced ultrasound and enhanced CT combined with tumor markers AFP and CA199 in the diagnosis of liver cancer were significantly higher than that of a single test.

**Conclusion:**

The combined detection of contrast-enhanced ultrasound and enhanced CT, AFP, and CA199 significantly improved the sensitivity and accuracy of liver cancer diagnosis. It has a significant effect on the early diagnosis of liver cancer and can be used as an important means of early screening.

## 1. Introduction

Liver cancer is a common clinical malignant tumor, which mostly develops from viral cirrhosis and hepatitis B. It has the characteristics of insidious onset, rapid progress, high metastasis rate, high fatality rate, and poor prognosis [1]. Most patients with benign liver disease have no specific symptoms and are easily ignored by patients. As the disease progresses, patients may experience pain, discomfort, and lumps in the upper right abdomen. When the patient went to the hospital for examination, it was obvious that there was a hard lump on the surface of the liver. And the mass can move up and down with breathing and eventually can progress to malignant tumors [2, 3]. Surgical treatment is a common clinical treatment method for liver cancer [4]. Therefore, the early screening and diagnosis of tumors are of great significance for the targeted therapy of patients and the improvement of patient prognosis.

Liver biopsy is the “gold standard” for the clinical diagnosis of liver cancer, but this method has certain limitations. It not only causes some trauma to patients, but not all patients can apply [5]. Therefore, finding an accurate and efficient noninvasive detection method has become the goal of many medical workers. Enhanced CT and contrast-enhanced ultrasound are common imaging diagnostic methods [6, 7]. Enhanced CT not only has higher tissue resolution and spatial resolution, but also can observe tiny lesions. It can also reflect the dynamic circulation process of the contrast agent in the liver, increase the positive detection rate of liver cancer, and reduce missed diagnosis [8]. Contrast-enhanced ultrasound technology is simple to operate and low in price. Microvascular technology can also be used to observe the blood flow status of the lesion, and the diagnosis accuracy rate is high [9].

It has been found that a variety of tumor markers are abnormally expressed in malignant tumors. They are a kind of biochemical substance produced by tumor cell proliferation or the host's response to tumor [10, 11]. It can be used as an important indicator for the early diagnosis of the disease by detecting the content of tumor markers in the patient's blood and tissues to determine the degree of disease progression. Among them, alpha-fetoprotein (AFP) and carbohydrate antigen 199 (CA199) are highly expressed in the serum of liver cancer patients [12, 13]. AFP is a highly specific serum glycoprotein. And the positive detection rate can be used as an important indicator of the clinical diagnosis of liver cancer [14]. CA199 is also a glycoprotein. Under normal circumstances, serum CA199 levels in patients with gastrointestinal tumors will increase significantly [15]. Therefore, if the patient's serum CA199 level is significantly increased, it means that they may have pancreatitis, liver cirrhosis, diabetes, and other diseases [16]. In addition, it has been reported that the combined detection of contrast-enhanced ultrasound and enhanced CT, AFP, and CA199 can effectively improve the sensitivity and specificity of liver cancer diagnosis [17–19], which is conducive to early screening of disease.

In this study, 256 liver cancer patients were compared with 110 patients with benign liver disease and 50 healthy people. This study aims to analyze the application value of contrast-enhanced ultrasound and enhanced CT and tumor markers AFP and CA199 in the clinical diagnosis of liver cancer.

## 2. Materials and Methods

### 2.1. Patients

This study is a retrospective study. 256 liver cancer patients from March 2017 to October 2020 were selected (liver cancer group). All patients were diagnosed pathologically, including 165 males and 91 females. The average age is 56.5 ± 9.5 years. 110 patients with benign liver lesions were selected into the benign lesion group. Among them, 71 were males and 39 were females, aged 57.5 ± 9.0 years old. 50 healthy people who have undergone physical examination were selected as the control group. There were 32 males and 18 females, aged 56 ± 9.0 years old. This study was approved by the Ethics Committee of People's Hospital of Rizhao. There was no statistically significant difference in general information among the three groups.

### 2.2. Inclusion and Exclusion Criteria

  Inclusion criteria: (1) meet the “Standards for Diagnosis and Treatment of Primary Liver Cancer” [20]; (2) patients who voluntarily sign informed consent forms; (3) patients who have not undergone surgery before participating in the study; and (4) patients who have complete clinical case data.
  Exclusion criteria: (1) patients with other malignant tumors; (2) patients with mental illness and those who do not cooperate with relevant examinations; (3) patients with blood system diseases; and (4) patients with allergies to the drugs used in this study.

### 2.3. Contrast-Enhanced Ultrasound

Both groups of patients used PHILIPSEPIQ5 color ultrasound diagnostic apparatus for contrast-enhanced ultrasound examination with a probe frequency of 5 MHz. Before the examination, the patient fasted for 8 hours and took the left side lying position. After the coupling agent was applied to the abdomen, the liver was thoroughly examined with conventional ultrasound. The location, size, shape, edge echo, internal echo, relationship with surrounding organs, and lymph nodes of the lesion were observed. Then, color Doppler mode was used to observe the blood flow in and around the lesion. The cut surface that is least affected by the patient's breathing can clearly show the lesion was selected. And the probe position was fixed. 2.4 mL of Sonovir (Bracco Imaging B.V.); contrast medium suspension was injected through superficial venous puncture of the patient's left elbow, and then 5 mL of normal saline was added. The arterial phase, portal phase, and delayed images were acquired at 30 s, 60 s, and 90 s after injection, respectively. After diagnosis, all patients received conventional surgical treatment. And the postoperative pathological examination results were recorded. An example of pathological examination is shown in Figure 1.

### 2.4. Enhanced CT Examination

Both groups of patients used the 64-slice spiral CT machine produced by GE in the USA for enhanced CT examination. First, a plain scan was performed on the patient's upper abdomen with a voltage of 120 kV, a tube current of 600 mA, and an interval of 0.965. A biphasic (arterial phase and portal vein phase) dynamic enhancement scan was performed on the patient's upper abdomen. 100 mL of iopromide injection (approval number J20100030, Guangzhou Branch of Bayer Healthcare Co., Ltd.) was injected into the patient's cubital vein at a rate of 3 mL/s. At 30 s and 60 s after the start of the contrast agent injection, the patient was instructed to hold his breath and scan in the arterial phase and portal vein phase. The patient's CT image was reconstructed. All data are reconstructed with 2 mm layer thickness and 1 mm interval, and then transferred to the background workstation. The incoming images are processed accordingly.

### 2.5. AFP and CA199 Detection

5 mL of fasting cubital venous blood was centrifuged at 3000 r/min (centrifugal radius 15 cm) for 10 min. And the upper serum was separated. After standing for 6 hours, the ADVIA Centaur XP automatic chemiluminescence immunoassay analyzer produced by Siemens was used for AFP and CA199 detection. The experiment was performed using Siemens kits and in strict accordance with the instructions. The test result is compared with the normal value of the index test. If the sample value is higher than the normal value, it is positive. If it is lower than the normal value, it is negative. The normal ranges of various indicators are as follows: AFP: 0 ng/mL∼25 ng/mL; CA199: 0 *μ*g/mL∼39 *μ*g/mL.

### 2.6. Observation Indicators

The contents of AFP and CA199 in the three groups were compared. The sensitivity, specificity, and accuracy of AFP and CA199 in the diagnosis of liver cancer were compared. With surgical pathological tissue examination or immunological diagnosis results as the gold standard, the diagnostic value of the combination of contrast-enhanced ultrasound and enhanced CT, AFP, and CA199 for liver cancer was compared. In the single test method, a positive judgment is liver cancer, and a negative judgment is a benign lesion. In the case of combined detection, if all 4 testing methods are negative, it is considered to be a benign lesion. If any test method is positive, it is judged as liver cancer. All images were read by two senior radiologists. It is considered valid when the conclusions are consistent. When the conclusions are inconsistent, other doctors were jointed or discussed together to reach a consensus as the final diagnosis.

  Sensitivity calculation method: true-positive number/(true-positive number + false-negative number) × 100%.
  Specificity calculation method: true-negative number/(true-negative number + false-positive number) × 100%.
  Accuracy calculation method: (true-positive number + true-negative number)/total number of cases × 100%.

### 2.7. Statistical Analysis

All experiments were repeated 3 times. Statistical analysis was performed using SPSS 23.0 software. The measurement data are expressed by $\bar{x}\pm s$, and the counting data are expressed as a ratio (%). The *X*^2^ test is used to analyze the data. Receiver operating curve (ROC) was drawn to obtain the area under the curve (AUC). The diagnostic value of AFP and CA199 combined contrast-enhanced ultrasound and enhanced CT detection for liver cancer was calculated. The difference was statistically significant at *P* < 0.05.

## 3. Results

### 3.1. The Diagnostic Value of Contrast-Enhanced Ultrasound and Enhanced CT for Liver Cancer Is Compared

For liver cancer, contrast-enhanced ultrasound diagnosed 227 positive cases and 96 negative cases (Table 1). Enhanced CT diagnosed 201 positive cases and 81 negative cases (Table 1). The above results indicate that the detection rate of contrast-enhanced ultrasound is higher than that of enhanced CT.

### 3.2. Comparison of Ultrasound Characteristics between Patients with Liver Cancer and Benign Liver Lesions

The proportion of liver cancer patients in terms of tumor boundary, echo, morphology, aspect ratio, blood flow signal, and lymph node metastasis were significantly higher than that of patients with benign lesions (*P* < 0.01, Table 2).

### 3.3. Contrast-Enhanced Ultrasound Images

Figures 2 and 3, respectively, show the liver, gallbladder, pancreas, spleen, kidney, and other parts of the patient.  Figure 2 shows liver cancer at stage I. The patient's liver section was slightly larger. The surface of the envelope was not smooth. The echo in the liver was thickened and enhanced, and the distribution was uneven. The structure of the intrahepatic duct was blurred, and the echo was abnormal. The inner edge was clear. The wall was thin, and the rear echo was enhanced. The shape and size of the gallbladder section were normal. No obvious abnormal echo was found. The shape and size of the pancreas were normal, and the pancreatic duct was not significantly expanded. Due to the influence of gas, the tail display was not clear. The spleen and kidneys were normal.  Figure 3 shows liver cancer in stage III. The patient's liver slice had abnormal morphology. The surface of the envelope was not smooth. Echoes in the liver were enhanced and thickened, and the distribution was uneven. Tumors can be found in the liver and vary in size and shape. The internal echo was low, and the edges were not clear. The tail of the pancreas was unclear. The gallbladder, spleen, and kidneys were all normal.

### 3.4. Enhanced CT Image

An example of enhanced CT image for liver cancer patients is shown in Figure 4.  Figure 4(a) shows the liver cancer at stage I. The shape and size of the patient's liver were normal. The right lobe of the liver was round and slightly low-density shadow, and the boundary was unclear.  Figure 4(b) shows liver cancer in stage II. Circular low-density shadow can be found in the patient's liver. And the boundary was not clear.  Figure 4(c) shows liver cancer in stage III. The patient's liver was full, and the edges were not smooth. Large areas of low-density shadows were found in the liver.  Figure 4(d) shows the liver cancer in stage III. The patient's liver was morphologically abnormal. Multiple low-density shadows and high-density deposits can be found in the liver. The boundary of the lesion was unclear.

### 3.5. Comparison of Serum AFP and CA199 Levels in the Three Groups

Serum levels of AFP and CA199 in the liver cancer group were 191.43 ± 21.66 ng/mL and 87.57 ± 11.45 *μ*g/mL, respectively. In addition, the levels of serum AFP and CA199 in the liver cancer group were significantly higher than those in the benign lesion group and the control group (*P* < 0.01, Figures 5 and 6).

ROC curve of AFP and CA199 combined with contrast-enhanced ultrasound and enhanced CT for the diagnosis of liver cancer.

The area under the ROC curve for the diagnosis of liver cancer by CA199 was 0.724 (0.563∼0.907), and the best cutoff value was 91.66 (Figure 7). The area under the ROC curve for the diagnosis of liver cancer by AFP was 0.747 (0.581∼0.931), and the best cutoff value was 187.65 (Figure 7). The area under the ROC curve of AFP and CA199 combined with contrast-enhanced ultrasound and enhanced CT in the diagnosis of liver cancer is 0.962 (0.896∼0.997, Figure 7).

### 3.6. The Diagnostic Value of Contrast-Enhanced Ultrasound and Enhanced CT Combined with Tumor Markers AFP and CA199 in Liver Cancer Is Compared

The sensitivity of combined detection for liver cancer was 96.88%. The specificity was 91.82%, and the accuracy was 95.36%. The positive prediction rate was 96.50%, and the negative prediction rate was 92.66%. Sensitivity, specificity, accuracy, positive prediction rate, and negative prediction rate were all higher than individual trials (Table 3). The sensitivity, accuracy rate, and negative prediction rate were significantly higher than the single tests (*P* < 0.05, Table 3).

## 4. Discussion

In recent years, with the changes in people's living standards and eating habits, the incidence of liver cancer has increased year by year. It mostly occurs in the elderly and is related to factors such as liver cirrhosis, viral hepatitis, and carcinogens. Liver cancer patients are present with abdominal distension, weight loss, and liver pain. Liver cancer has the characteristics of high degree of malignancy and great harm [21]. Early liver cancer has no obvious clinical symptoms, and early liver cancer is not easy to attract attention [22]. Therefore, the diagnosis of liver cancer is difficult. With the development of the disease, the fibrous tissue of the liver increases, which evolves into liver focal nodular hyperplasia—cirrhosis—liver cancer. Hypofunction of liver will seriously shorten the survival time of patients and even endanger the life safety of patients [23]. Therefore, the early diagnosis and treatment of liver cancer are very important for prolonging the survival time and improving the life quality of patients. Pathological diagnosis is the gold standard for clinical diagnosis of liver cancer [24]. However, pathological diagnosis will cause certain skin trauma to the patient. At the same time, needle tract bleeding is prone to occur. These limitations make it difficult for many patients to accept. On the other hand, the sample size of liver biopsy is small and cannot fully reflect the pathological conditions of the liver [25]. If the liver lesions are unevenly distributed, the diagnosis may be wrong.

As we all know, the content of serum tumor markers will change with the continuous development of the disease. The detection of serum tumor markers helps to detect abnormalities in the body as soon as possible and improve the early diagnosis rate of tumors [26]. AFP and CA199 are commonly used tumor markers for the diagnosis of liver cancer. Although the detection of the two marker levels is simple, the detection sensitivity and specificity are not high [27, 28]. Therefore, missed diagnosis can easily occur because these two serum markers are highly expressed not only in liver cancer patients, but also in many other malignant tumors. This brings difficulties to the differential diagnosis of liver cancer. This study showed that the levels of AFP and CA199 in the liver cancer group were higher than those in the benign liver disease group and the control group. The proliferation of liver cancer cells stimulates the expression of AFP and CA199 in serum, leading to a significant increase in the levels of AFP and CA199. However, patients with benign lesions only show inflammation. Although the levels of AFP and CA199 have also increased, their levels are much lower than those of the liver cancer group.

In recent years, imaging technology has developed rapidly in the medical field. It plays a key role in the early screening of malignant tumors and provides an important reference for rationally formulating surgical plans and prognostic effects [29, 30]. Contrast-enhanced ultrasound and enhanced CT are important imaging methods for the clinical diagnosis of liver cancer. Enhanced CT can clearly observe small lesions and can also better reflect blood flow through the use of contrast agents. It can also prevent image artifacts caused by normal breathing and provide imaging evidence for the clinical diagnosis of liver cancer [31]. However, the presence of ionizing radiation in this test will cause a certain degree of harm to the patient's body. At the same time, the blood supply of some patients with benign lesions and some liver cancer patients is almost the same, which is easy to cause misdiagnosis or missed diagnosis [32]. Contrast-enhanced ultrasound technology is a new type of ultrasound imaging detection technology. The contrast agent contains tiny bubbles to enhance the scattered echo, thereby improving the accuracy and sensitivity of disease diagnosis [33]. It not only has the ability of ordinary two-dimensional ultrasound to diagnose tumor echo, morphology, boundary, and other nonquantifiable indicators [34], but also increases the qualitative and quantitative information of blood perfusion. Therefore, the contrast-enhanced ultrasound technology can show the differences between different liver lesions more intuitively and in detail [35]. In addition, the nonradiation, noninvasiveness, and high-cost performance of this technology make it popular with patients and clinicians [36]. In this study, the detection rate of contrast-enhanced ultrasound was significantly higher than that of enhanced CT. Although enhanced CT has high tissue resolution and can show small lesions, it is easily confused with liver hemangioma, liver cyst, and other diseases, which increases the misdiagnosis rate [37]. The time of contrast-enhanced ultrasound examination is longer than that of enhanced CT, which can make the blood vessels and small lesions more clearly and accurately displayed [38].

This study found that the combined detection of contrast-enhanced ultrasound and enhanced CT, AFP, and CA199 has a high diagnostic value for the early diagnosis of liver cancer. The sensitivity and accuracy of combined detection for diagnosing liver cancer were 96.88% and 95.36%, which were significantly higher than single detection. It is suggested that the diagnostic value of combined detection in liver cancer is better than single detection, which is helpful for the early clinical diagnosis of liver cancer. Combined detection can better make up for the shortcomings of single index detection in the diagnosis of liver cancer and improve the accuracy of diagnosis. However, the sample of this study is still relatively small. In the future, we need to continue to expand the sample size to further verify our conclusions.

## 5. Conclusion

In summary, the combined detection effect is significant, improves the sensitivity and accuracy of diagnosis, and is beneficial to the early diagnosis of liver cancer. Therefore, combined detection can be used as an auxiliary form of clinical screening for early liver cancer and provide a reference basis for clinicians to formulate a reasonable plan and prognosis.

## Figures and Tables

**Figure 1:** The example diagram of pathological examination. (a) Hepatocellular carcinoma (grade II). The tumor volume is 1.9*∗*1.3*∗*0.4 cm. Most of the tumor cells are located in the bile duct without invading the liver capsule. The surrounding liver tissue showed chronic inflammation (G3S4), but no tumor was found at the surgical margin of nodular cirrhosis. (b) Moderately differentiated hepatocellular carcinoma. The tumor volume is 2.5*∗*2.5*∗*2 cm, without invasion of the capsule. No tumor thrombus was found in the vessel, and the small nerve bundles were not involved. Cancer was found at the surgical margin. (c) Moderately differentiated hepatocellular carcinoma. The tumor volume is 13.5*∗*10.5*∗*5.8 cm, and it did not invade the liver capsule. The surrounding liver tissue showed changes in liver cirrhosis, and no cancer was found at the surgical margin. (d) Liver nodule. The proliferation of hepatocytes is active under the microscope. And the hepatic cord is widened.

**Figure 2:** The picture of contrast-enhanced ultrasound for liver cancer at stage I.

**Figure 3:** The picture of contrast-enhanced ultrasound for liver cancer at stage III.

**Figure 4:** Enhanced CT image.

**Figure 5:** The serum level of AFP was compared between the liver cancer group (*n* = 256) and the control group (*n* = 50) or benign lesion group (*n* = 110). *P* < 0.05.

**Figure 6:** The serum level of CA199 was compared between the liver cancer group (*n* = 256) and the control group (*n* = 50) or benign lesion group (*n* = 110). *P* < 0.05.

**Figure 7:** ROC curve of AFP and CA199 combined with contrast-enhanced ultrasound and enhanced CT in diagnosing liver cancer (*n* = 256).

**Table 1:** Comparison of the diagnostic value of contrast-enhanced ultrasound and enhanced CT for liver cancer (*n*).

Features	Contrast-enhanced ultrasound		Enhanced CT		Total
	Positive	Negative	Positive	Negative	
Positive	227	29	201	55	256
Negative	14	96	24	86	110
Total	241	125	225	141	366

**Table 2:** Comparison of ultrasound characteristics between patients with liver cancer and benign liver lesions (*n*).

Ultrasound characteristics		Liver cancer (*n* = 256)	Benign lesions (*n* = 110)	*X* ^2^	*P*
Location	Middle-upper	143	69	1.489	>0.05
	Bottom	113	41		

Boundary	Distinct	84	73	35.358	<0.01^*∗∗*^
	Blurry	172	37		

Echo	Symmetrical	68	66	37.067	<0.01^*∗∗*^
	Unevenness	188	44		

Morphology	Regular	91	75	33.063	<0.01^*∗∗*^
	Irregularity	165	35		

Aspect ratio	>1	157	37	23.686	<0.01^*∗∗*^
	≤1	99	73		

Blood flow signal	0∼1	61	82	83.135	<0.01^*∗∗*^
	2∼3	195	28		

Lymph node metastasis	No	101	27	7.519	<0.01^*∗∗*^
	Yes	155	83		

^*∗∗*^ *P* < 0.01.

**Table 3:** Comparison of the diagnostic value of contrast-enhanced ultrasound and enhanced CT combined with tumor markers AFP and CA199 in liver cancer.

Method	Sensitivity	Specificity	Accuracy	Positive rate	Negative rate
Contrast-enhanced ultrasound	88.67 (227/256)	87.27 (96/110)	88.25 (323/366)	94.19 (227/241)	76.80 (96/125)
Enhanced CT	78.52 (201/256)	78.18 (86/110)	78.42 (287/366)	89.33 (201/225)	60.99 (86/141)
AFP	77.73 (199/256)	80.00 (88/110)	78.42 (287/366)	90.05 (199/221)	60.69 (88/145)
CA199	78.13 (200/256)	70.00 (77/110)	75.68 (277/366)	85.84 (200/233)	57.89 (77/133)
Combined detection	96.88 (248/256)	91.82 (101/110)	95.36 (349/366)	96.50 (248/257)	92.66 (101/109)
*X* ^2^	7.614	1.335	6.143	2.012	10.467
*P* value	<0.05^*∗*^	>0.05	<0.05^*∗*^	>0.05	<0.05^*∗*^

^*∗*^ *P* < 0.05.

## Data Availability

Data to support the findings of this study are available on reasonable request from the corresponding author.

## References

[1] Tellapuri S., Sutphin P. D., Beg M. S., Singal A. G., Kalva S. P. (2018). Staging systems of hepatocellular carcinoma: a review. *Indian Journal of Gastroenterology*.

[2] Cai M.-J., Cui Y., Fang M. (2019). Inhibition of PSMD4 blocks the tumorigenesis of hepatocellular carcinoma. *Gene*.

[3] Li L., Gou C.-Y., Li J.-Y., Achakzai R., Li X.-H. (2016). Cancer of the Liver Italian Program score helps identify potential candidates for transarterial chemoembolization in patients with Barcelona Clinic Liver Cancer stage C. *Hepatobiliary and Pancreatic Diseases International*.

[4] Tangoku A. (2017). Team Approach for surgical treatment, present status and perspective. *Nihon Geka Gakkai Zasshi*.

[5] Arafah M., Kfoury H. (2017). Radiological tests versus pathological diagnostics: complimentary or antagonistic relationship? The experience of a tertiary hospital. *Indian Journal of Pathology & Microbiology*.

[6] Luedemann W. M., Geisel D., Gebauer B. (2020). Comparing HCC arterial tumour vascularisation on baseline imaging and after lipiodol cTACE: how do estimations of enhancing tumour volumes differ on contrast-enhanced MR and CT?. *European Radiology*.

[7] Kim T. K., Noh S. Y., Wilson S. R. (2017). Contrast-enhanced ultrasound (CEUS) liver imaging reporting and data system (LI-RADS) 2017-a review of important differences compared to the CT/MRI system. *Clinical and Molecular Hepatology*.

[8] Minami Y., Kudo M. (2015). Imaging modalities for assessment of treatment response to nonsurgical hepatocellular carcinoma therapy: contrast-enhanced US, CT, and MRI. *Liver Cancer*.

[9] Kim T.-H., Yoon J. H., Lee J. M. (2019). Emerging role of hepatobiliary magnetic resonance contrast media and contrast-enhanced ultrasound for noninvasive diagnosis of hepatocellular carcinoma: emphasis on recent updates in major guidelines. *Korean Journal of Radiology*.

[10] Sauerbrei W., Taube S. E., McShane L. M., Cavenagh M. M., Altman D. G. (2018). Reporting recommendations for tumor marker prognostic studies (REMARK): an abridged explanation and elaboration. *Journal of the National Cancer Institute: Journal of the National Cancer Institute*.

[11] Nishida N., Kudo M. (2017). Oncogenic signal and tumor microenvironment in hepatocellular carcinoma. *Oncology*.

[12] Park S. J., Jang J. Y., Jeong S. W. (2017). Usefulness of AFP, AFP-L3, and PIVKA-II, and their combinations in diagnosing hepatocellular carcinoma. *Medicine*.

[13] Scarà S., Bottoni P., Scatena R. (2015). CA 19-9: biochemical and clinical aspects. *Advances in Cancer Biomarkers*.

[14] Qi F., Zhou A., Yan L. (2020). The diagnostic value of PIVKA-II, AFP, AFP-L3, CEA, and their combinations in primary and metastatic hepatocellular carcinoma. *Journal of Clinical Laboratory Analysis*.

[15] Ammer-Herrmenau C., Neesse A. (2020). CA19-9: mehr als nur ein Biomarker?. *Zeitschrift für Gastroenterologie*.

[16] Luo G., Fan Z., Cheng H. (2018). New observations on the utility of CA19-9 as a biomarker in Lewis negative patients with pancreatic cancer. *Pancreatology*.

[17] Edoo M. I. A., Chutturghoon V. K., Wusu-Ansah G. K. (2019). Serum biomarkers AFP, CEA and CA19-9 combined detection for early diagnosis of hepatocellular carcinoma. *Iranian Journal of Public Health*.

[18] Huang X., Li J., Wang F., Hao M. (2018). CT combined with tumor markers in the diagnosis and prognosis of hepatocellular carcinoma. *Journal of B.U.ON.: Official Journal of the Balkan Union of Oncology*.

[19] Minami Y., Nishida N., Kudo M. (2014). Therapeutic response assessment of RFA for HCC: contrast-enhanced US, CT and MRI. *World Journal of Gastroenterology*.

[20] Zhou J., Sun H.-C., Wang Z. (2018). Guidelines for diagnosis and treatment of primary liver cancer in China (2017 edition). *Liver Cancer*.

[21] Kudo M. (2015). Chronic liver diseases and liver cancer: an update in 2015. *Digestive Diseases*.

[22] Hansen P. D., Cassera M. A., Wolf R. F. (2015). Ablative technologies for hepatocellular, cholangiocarcinoma, and metastatic colorectal cancer of the liver. *Surgical Oncology Clinics of North America*.

[23] Lujambio A., Villanueva A. (2015). The usual SASPects of liver cancer. *Aging*.

[24] Jabbour T. E., Lagana S. M., Lee H. (2019). Update on hepatocellular carcinoma: pathologists’ review. *World Journal of Gastroenterology*.

[25] Ozer Etik D., Suna N., Boyacioglu A. S. (2017). Management of hepatocellular carcinoma: prevention, surveillance, diagnosis, and staging. *Exp Clin Transplant*.

[26] Juntermanns B., Kaiser G. M., Itani Gutierrez S. (2018). CA19-9 beim intrahepatischen Cholangiokarzinom. *Chirurg, Der*.

[27] Lu Q., Li J., Cao H., Lv C., Wang X., Cao S. (2020). Comparison of diagnostic accuracy of Midkine and AFP for detecting hepatocellular carcinoma: a systematic review and meta-analysis. *Bioscience Reports*.

[28] Arias-Flórez J. S., Martínez-Delgado A. M., Alarcón-Tarazona M. L., Insuasty-Enriquez J. S., Díaz-Martínez L. A. (2018). Rendimiento diagnóstico de marcadores tumorales séricos convencionales en pacientes con sospecha clínica de cáncer primario metastásico a hígado. *Revista Medica de Chile*.

[29] Jiang H.-Y., Chen J., Xia C.-C., Cao L.-K., Duan T., Song B. (2018). Noninvasive imaging of hepatocellular carcinoma: from diagnosis to prognosis. *World Journal of Gastroenterology*.

[30] Kim T.-H., Kim S. Y., Tang A., Lee J. M. (2019). Comparison of international guidelines for noninvasive diagnosis of hepatocellular carcinoma: 2018 update. *Clinical and Molecular Hepatology*.

[31] Coskun M. (2017). Hepatocellular carcinoma in the cirrhotic liver: evaluation using computed tomography and magnetic resonance imaging. *Experimental and Clinical Transplantation: Official Journal of the Middle East Society for Organ Transplantation*.

[32] Li J., Li X., Weng J. (2018). Gd-EOB-DTPA dynamic contrast-enhanced magnetic resonance imaging is more effective than enhanced 64-slice CT for the detection of small lesions in patients with hepatocellular carcinoma. *Medicine*.

[33] Tanaka H. (2020). Current role of ultrasound in the diagnosis of hepatocellular carcinoma. *Journal of Medical Ultrasonics*.

[34] Lencioni R., Piscaglia F., Bolondi L. (2008). Contrast-enhanced ultrasound in the diagnosis of hepatocellular carcinoma. *Journal of Hepatology*.

[35] Guo L. H., Xu H. X. (2015). Contrast-enhanced ultrasound in the diagnosis of hepatocellular carcinoma and intrahepatic cholangiocarcinoma: controversy over the ASSLD guideline. *BioMed Research International*.

[36] McGillen K. L., Zaidi S., Ahmed A., Harter S., Yee N. S. (2020). Contrast-enhanced ultrasonography for screening and diagnosis of hepatocellular carcinoma: a case series and review of the literature. *Medicine*.

[37] Maiwald B., Lobsien D., Kahn T., Stumpp P. (2014). Is 3-Tesla Gd-EOB-DTPA-enhanced MRI with diffusion-weighted imaging superior to 64-slice contrast-enhanced CT for the diagnosis of hepatocellular carcinoma?. *PLoS One*.

[38] Xu R., Wang J., Huang X. (2019). Clinical value of spectral CT imaging combined with AFP in identifying liver cancer and hepatic focal nodular hyperplasia. *Journal of B.U.ON.: Official Journal of the Balkan Union of Oncology*.

